# 16SrDNA-Based Detection Technology in Patients with Chronic Pharyngitis to Analyze the Distribution Characteristics of Pharyngeal Bacteria

**DOI:** 10.1155/2022/5186991

**Published:** 2022-03-11

**Authors:** Yage Shen, Chunhan Liu, Jiao Luo, Jianchao Wang, Di Zhang

**Affiliations:** ^1^The Affiliated Hospital of Hebei University/College of Clinical Medicine, Baoding 071000, China; ^2^Department of Otolaryngology, The Third People's Hospital of Shenzhen (The Second Affiliated Hospital of Southern University of Science and Technology), Shenzhen 518000, China; ^3^Vertigo Clinic, The Third People's Hospital of Shenzhen (The Second Affiliated Hospital of Southern University of Science and Technology), Shenzhen 518000, China

## Abstract

In order to analyze the distribution characteristics of pharyngeal bacteria in patients with chronic pharyngitis (CP) by 16SrDNA-based detection technology, a prospective study is conducted to collect pharyngeal secretion samples from patients diagnosed with CP who are admitted to the Otorhinolaryngology Department of The Third People's Hospital of Shenzhen from May 2021 to September 2021. Among them, 11 cases are chronic simple pharyngitis (CSP), 11 cases are chronic hypertrophic pharyngitis (CHP), and 8 cases are healthy subjects. All samples are detected by the 16SrDNA technique and analyzed by bioinformatics. 55724.64 ± 1772.80, 53697.73 ± 2252.19, and 55177.5 ± 1661.80 optimized sequences are obtained by 16SrDNA sequencing. The *α* diversity analysis of pharyngeal microflora showed that the abundance index SOBS of pharyngeal microflora is upregulated in patients with CHP compared with normal controls (NC), but the diversity index of pharyngeal bacteria in the three groups is not significantly changed, indicating that the abundance of pharyngeal bacteria in the CHP group is increased. The *β* diversity analysis of pharyngeal microflora showed that the three groups are similar in structure and composition, and there is no significant statistical difference. The structural difference analysis of pharyngeal flora combined with LEfSe difference analysis showed that at the phylum level, the relative abundance of Spirochaetes and Synergistetes in the CHP group is significantly higher than that in the CSP group. At the genus level, the relative abundance of opportunistic pathogens such as Selenomonas and *Campylobacter* increased significantly in the CSP group. The relative abundance of *Escherichia*, Mycoplasma, and Porphyromonas are significantly increased in the CHP group. The abundance of beneficial symbiotic bacteria decreased significantly in patients with CP. The pharyngitis of patients with CP is characterized by an increase in the abundance of pharyngitis, changes in the structure of pharyngitis, a decline in the symbiotic beneficial bacteria, and an increase in the content of opportunistic pathogens, which may be closely related to the onset and development of CP.

## 1. Introduction

Chronic pharyngitis (CP) is a common disease in otorhinolaryngology characterized by chronic inflammation of the mucosa, submucosa, and lymphocytes. According to pharyngeal manifestations, chronic simple pharyngitis (CSP) and chronic hypertrophic pharyngitis (CHP) can be divided into two clinical case types. Statistically, CP accounts for 10–20% of pharyngeal diseases and 12–14% of otorhinolaryngology diseases, with the incidence increasing year by year [1, 2]. With the rapid development of industrialization, the incidence of chronic pharyngitis in high PM2.5 areas is much higher than that in mildly polluted areas [3]. CP is characterized by high incidence and low cure rate, which not only reduces the quality of life of patients but also increases the difficulty of clinical standard medication and even causes the abuse of antibiotics [4].

CP is a multifactorial disease, including chronic infectious factors, noninfectious factors, physical and chemical factors, stimulation, occupational factors, and lifestyle [5, 6]. Currently, microbiome as a driving factor involved in the pathogenesis of chronic mucosal inflammatory diseases has gradually attracted attention [7–11]. Some scholars determined the relatively simple bacterial community composition of CP through traditional bacterial culture identification methods, and *α*-hemolytic streptococcus ranked first among many strains [12, 13]. However, the identification results are easily affected by different culture times and growth environment requirements. Compared with traditional culture technology, second-generation sequencing (16SrDNA detection technology) is a more sensitive microbiome detection method, which can display the distribution of microorganisms in the pharynx more comprehensively. At present, in otorhinolaryngology-related diseases, a complicated bacterial spectrum such as rhinosinusitis [7, 8], otitis media [9], and allergic rhinitis [10, 11] has been identified by second-generation sequencing. In this study, the diversity and difference in pharyngitis bacteria in patients with CP and healthy subjects are analyzed by the 16SrDNA sequencing method, and the correlation between the distribution of bacteria and CP is explored, aiming to provide new ideas for the clinical treatment of CP.

## 2. Clinical Protocol

### 2.1. Experimental Objects and Grouping

A total of 22 patients diagnosed with CP who visited the Otorhinolaryngology Department of The Third People's Hospital of Shenzhen from May 2021 to September 2021 are collected. Among them, there are 11 CSP, 11 CHP, and 8 healthy volunteers. The main symptoms of CP patients include pharyngeal foreign body sensation, dry pharynx, pharyngeal itching, frequent throat clearing, cough, phlegm, pharyngeal pain, and other pharyngeal discomfort symptoms.

### 2.2. Inclusion Criteria

Inclusion criteria were defined as follows:

1. It conforms to the diagnostic criteria of CSP and CHP in the Practice of Otolaryngology-Head and Neck Surgery (2nd edition)
2. Age ≥18 years old
3. Informed consent and sign a notice, and volunteer to provide clinical sample collection
4. There are no obvious neoorganisms in the pharynx and larynx under electronic laryngoscopy
5. No obvious bacterial formation is found in the general bacterial culture in the laboratory

### 2.3. Exclusion Criteria

Exclusion criteria were defined as follows:

1. Chronic inflammation of the upper respiratory tract: rhinitis, sinusitis, nasopharyngitis; tonsillitis, adenoid hypertrophy (residual)
2. Adjacent organs and disease stimulation: oral diseases: dental caries, periodontitis; esophageal and gastric diseases: reflux esophagitis, reflux gastritis; trachea and lung diseases: chronic bronchitis, chronic pneumonia
3. Allergic diseases: allergic rhinitis and allergic pharyngitis
4. Other diseases caused by pharyngeal discomfort symptoms are as follows: esophageal cancer, styloid syndrome, hyoid syndrome, pharyngeal syndrome, pharyngeal *tuberculosis*
5. Chemical or physical therapy, such as antibiotics, vitamins, atomization, microwave, and laser, is used two weeks before the visit

### 2.4. Sample Collection

In a sterile dressing room, the patient is seated with his mouth open and his head tilted back. Samplers fixed their tongues with tongue spatters, and sterile flocking swabs are repeatedly wiped on the posterior and lateral pharyngeal walls three times. Pharyngeal secretions are collected and sent to Shenzhen BGI Co., LTD., for DNA extraction, sequencing, and analysis.

## 3. Pharyngeal Microflora Detection

### 3.1. 16SrDNA Sequencing

The V3–V4 region of the 16SrDNA gene is amplified by polymerase chain reaction (PCR) with sample DNA as a template. Then Agencourt AMPure XP magnetic beads are used to purify PCR products and dissolve them in the elution buffer to complete the construction of library. And Agilent 2100 Bioanalyzer is used to detect the fragment range and concentration of the library. Finally, the qualified libraries are sequenced using the Illumina HiSeq platform according to the inserted fragment size.

### 3.2. Bioinformatics Analysis

The original sequencing data are filtered to obtain high-quality clean data for analyses. Reads would be joined together into tags by overlap relations between reads, and tags with a similarity of above 97% would be grouped into operational taxonomic units (OTUs) and compared with the Greengenes database for taxonomic analysis, and community species annotation of phylum, class, order, family, genus, and species of each group of samples would be counted.

Statistical analysis and visualization of microbial community composition and structure are performed based on OTU and annotation results. Veen diagrams are drawn by R (V3.2.1) software to show the number of common and unique OTU in multiple samples, which can intuitively display the overlap of OTU between samples. The OTU accumulation curve is plotted to reflect the influence of sampled individuals on species diversity. Draw a dilution curve to determine the appropriate amount of sequencing for the sample. Mother (V.1.31.2) software is used for *α* diversity analysis, which reflects the diversity of species, community richness, and evenness within the ecosystem. The indexes of community richness mainly included the Chao1 index, the ACE index, and the SOBS index. Community diversity index includes the Shannon index and Simpson index. The test level *α* = 0.05 and *P* < 0.05 is considered statistically significant. *β* diversity is used to analyze the evolutionary relationship and abundance information of the three groups to compare the significant differences in the composition of microbial communities. QIIME (V1.80) software is used for principal coordinate analysis (PCoA) to show differences in community composition among the three groups of samples. The abscissa represents one principal component, the ordinate represents another, and the percentage represents the contribution value of the principal component to the sample difference. If the samples are closer to each other, the species composition and structure are more similar. Samples with high similarity in community composition tended to cluster together, while samples with great community differences tended to separate. R (V3.4.1) software is used to analyze differences between beta groups, and a box graph of the beta diversity index is drawn. The test level *α* = 0.05 and *P* < 0.05 is considered statistically significant.

R (V3.4.1) software is used to analyze the differences in the bacterial community structure of the three groups of samples, and the abundances of major species at phylum and genus levels and the analysis plots of different bacterial communities are drawn. The K-w rank sum test is used to analyze the differences between multiple groups, and the Wilcoxon rank sum test is used to analyze the differences between the two groups. The test level *α* = 0.05 and *P* < 0.05 is considered statistically significant.

The LEfSe software is used to calculate and draw the LDA graph to reflect the microbial communities with significant effects in the three groups of samples. When LDA ≥2.0, significant differences between species are considered.

SPSS 24.0 software is used to process the data. The Shapiro–Wilk test is used to test the normal distribution of continuous counting variables. The data of the normal distribution are expressed as *x* ± *S*, the multiple comparison *T* test is used, and the chi-square test is used for grade data. *P* < 0.05 indicates statistically significant differences.

## 4. Experimental Result

### 4.1. OTU Analysis of Pharyngeal Bacteria

There is no statistical difference in the number of optimized sequences of pharyngeal samples between the CHP, CSP, and normal control (NC) groups, as shown in Table 1. A total of 359 OTUs are obtained from 30 samples, including 265 OTUs. There are 25 OTUs in the CHP and NC groups, 24 OTUs in CHP and CSP, and 8 OTUs in CSP and NC groups. There are 25 OTUs in CHP, 7 OTU in CSP, and 4 OTUs in NC groups, respectively, as shown in Figure 1. The species accumulation curve tended to be flat with the increase of sample size. The dilution curve of pharyngeal flora tended to be flat with the increase of sequencing depth. This indicated that the amount of measured data is reasonable and basically reaches the sequencing depth, as shown in Figure 2.

### 4.2. *α* Diversity Analysis

The comparison of ACE, Chao, and SOBS indexes between CHP, CSP, and NC groups is statistically significant (*P* < 0.05). The SOBS index of CHP and NC groups is statistically significant (*P* < 0.05). There is no statistical significance in Shannon and Simpson index among the three groups, as shown in Figure 3. The index of ACE (a), Chao (b), SOBS (c, d), Shannon (e), and Simpson (f) comparison of pharyngeal microflora of the three groups are shown in Figure 3. *P* < 0.05 is considered a statistically significant difference.

### 4.3. Principal Coordinate Analysis and *β* Diversity Analysis

Principal coordinate analysis (PCoA) showed that the distribution of 30 samples is relatively concentrated, with no obvious separation tendency, indicating that the species composition of the flora had no statistical significance, as shown in Figure 4(a). By *β* diversity analysis, the mean and standard deviation of *β* diversity of each group are calculated. The box plot showed that there is no statistical difference in the species composition of the three groups, which is consistent with the above PCoA results, as shown in Figure 4(b).

### 4.4. Analysis of Differences in Bacterial Community Structure

At the phylum level, the pharyngeal flora consists of six phyla, including Bacteroidetes, Firmicutes, Fusobacteria, Proteobacteria, Actinobacteria, and TM7. Among them, Bacteroidetes and Firmicutes are obviously dominant, accounting for more than 60% of the total. Comparison of species structure among the three groups of samples showed that there are differences between Spirochaetes and Synergistetes, as shown in Figure 5(a). In addition, there is no significant change in phylum abundance between the CHP group and the CSP group compared with the NC group, as shown in Figure 5(c). Compared with the CHP group, the abundance of Spirochaetes and Synergistetes decreased in the CSP group, as shown in Figure 5(a). At the genus level, there are 17 genera in the pharynx, and the dominant bacteria are Prevotella, *Streptococcus*, and Veillonella, accounting for about 28%, 17%, and 10%, accounting for 55% of the 17 genera. The relative abundance of 14 genera in the three groups is statistically significant. Compared with the NC group, the abundance of Porphyromonas in the CSP group is decreased, while the abundance of *Campylobacter* and Selenomonas is increased. The abundance of Porphyromonas, Mycoplasma, and *Escherichia* increased in the CHP group. Compared with the CSP group, the abundance of Porphyromonas, Mycoplasma, and *Escherichia* increased in the CHP group. Compared with the CSP group, Desuliste, Desulphurobacte, *Campylobacter*, Olsenella, Acholeplasma, Filifactor, TG5, Porphyromonas, mycoplasma, *Escherichia*, *Treponema*, *Haemophilus*, and Johnsonell in the CHP group increased in abundance. Compared with the NC group, the abundance of the symbiotic beneficial bacteria Actinomyces decreased in the CHP and CSP groups, as shown in Figure 5(b) and Figure 5(d).  Table 2 shows the comparison of the relative abundance of pharyngeal flora at genus level.

### 4.5. LEfSe Difference Analysis

A LDA score absolute value ≥2.0 is considered a significantly difference. When the absolute value of theLDA score ≥2.0, there are 31 species with significant differences among the three groups, among which 5 species are enriched in the CSP group, namely, Selenomonas, Camplobacter, Campylobacteraceae, and Epsilonproteobacteria. 26 species are enriched in CHP group, that is, Acholeplasma, Synergistia, Dethiosulfovibrionaceae, TG5, Synergistales, Desulfobacteriale, Enterobacteriales, Mycoplasmatales, Mycoplasma, Mycoplasmataceae, Enterobacteriaceae, Tenericutes, Mollicutes, Acholeplasmataceae, Desulfobulbus, Desulfobulbaceae, Acholeplasmatales, *Escherichia*, Filifactor, Spirochaetes, Spirochaetaceae, Spirochaetale, *Treponema*, and Porphyromonadaceae. No significant enrichment is observed in the NC group, as shown in Figure 6.

## 5. Data Analysis and Discussion

In recent years, with the rapid development in the field of molecular biology, high-throughput sequencing technology based on the bacterial 16SrDNA gene has become the preferred method for identifying bacterial communities and species with reduced cost and iterative database updates. There is increasing evidence that diseases are not determined by pathogens alone, but by the complex balance between pathogens, resident microbiota, and host immune response.

In this study, the pharyngeal secretions samples of patients with CHP, CSP, and NC are detected by 16DSrDNA technology, and the differences among the three groups are preliminarily explored. 55724.64 ± 1772.80 optimized sequences of CHP are obtained. The optimal sequences are 53697.73 ± 2252.19 in CSP and 55177.50 ± 1661.80 in the NC group. According to the OTU accumulation curve and dilution curve of pharyngeal microflora, with the increase of sample size, the curve gradually flattened, and the OTU of sample microflora tended to be stable, indicating that the sample size of 30 cases is sufficient, the amount of measured data is reasonable, and the sequencing depth is basically reached.

By comparing pharyngeal microflora from multiple perspectives, *α* diversity analysis showed that the abundance of pharyngeal microflora increased in the CHP group, and there was no significant difference in diversity between the CSP and NC groups. PCoA and *β* difference analysis between groups showed that there is no significant difference in the composition of pharyngeal bacteria between patients with CP and healthy persons. These results indicated that the CHP group had more diverse pharyngeal microorganisms, and there is no sharp change in the pharyngitis individuals with different phenotypes.

From the comparison of phylum and genus, the abundance of Selenomonas and Camplobacter in the CSP group is higher than that in the NC group and the CHP group. The abundance of Spirochaetes, Synergistetes, Dialister, Desulfobacter, *Campylobacter*, Olsenella, ancholesteric, Filifactor, TG5, Porphyromonas, Mycoplasma, *Escherichia*, *Treponema*, *Haemophilus*, *Haemophilus*, and Johnsonella in the CHP group is higher than that in the NC group and CSP group. Combined with LEfSe difference analysis results, it is speculated that Spirochaetes, Synergistetes, Porphyromonas, Mycoplasma, and *Escherichia* might be markers of the CHP group. Selenomonas and Camplobacter may be the markers of CSP, suggesting that the changes of these bacterial communities are correlated with CP.

The respiratory tract of normal people is mainly colonized by Bacteroidetes, Firmicutes, Fusobacteria, Proteobacteria, and Actinobacteria. Different microenvironments, such as the nasal cavity, oral cavity, and lung, have different proportions of microbial communities. This study confirmed that the main dominant bacteria in normal pharyngeal flora are still Bacteroidetes and Firmicutes, but the abundance of Spirochaetes and Synergistetes increased significantly in the CHP group. Lipopolysaccharide, glycolipids, and membrane lipoproteins are the lipid-lipid interactions between Spirochaetes and their eukaryotic hosts. Lipoproteins are the most abundant proteins expressed in all Spirochaetes. It plays an important role in packaging, storage, and trans-membrane output from the ribosome to the cell surface. Compared with other proteins, it can promote inflammatory response and regulate immune response, assist pathogens to adhere to the host body, and realize the immune escape of Spirochaetes, thus causing persistent infection symptoms in the human body. Therefore, the increase of Spirochaetes may cause the disorder of pharyngeal flora in patients, and the abuse and misuse of antibiotics in clinical practice affect the immune function of the body and accelerate the disease process, resulting in prolonged CHP. Synergistetes exist widely in nature, and many kinds of bacteria have been isolated from the human oral cavity, intestinal tract, skin, and vagina, which are opportunistic pathogens. Synergistetes are closely related to oral periodontal inflammation and are also involved in more serious inflammation and tissue damage caused by oral microbial infections, such as necrotic ulcerative gingivitis. Studies have shown that Synergistetes have a negative effect on the downregulation of intestinal relative abundance in patients with Celiac disease, induce the production of protective IgM antibodies in the intestinal tract of patients with systemic lupus erythematosus, and play a positive role in protective humoral immune response. In addition, the relative abundance of Synergistetes is positively correlated with the intake of cholesterol, niacin, and selenium and negatively correlated with acetic acid and total short-chain fatty acids, further demonstrating the anti-inflammatory effect of Synergistetes. In this study, the relative abundance of Synergistetes in the CHP group, NC group, and CSP group decreased successively, suggesting that Synergistetes had a dynamic imbalance in the pharyngitis of patients with CP. One or more strains under the same phylum showed anti-inflammatory effects on CHP and CSP.

In addition to the homeostasis imbalance, another characteristic of CP is the increased relative abundance of opportunistic pathogens. In this study, the proportion of beneficial symbiotic bacteria, Actinomyces of Acfinobacteria and Prevotella of Bacteroidetes decreased in the pharynx of CP patients. If the addition of beneficial symbiotic bacteria prevents the adhesion and invasion of pathogens, cell integrity and permeability can be controlled, and then the interaction with the human epithelial surface can reduce the inflammatory response of the host, and the possibility of disease can be greatly reduced. Previous studies have shown that administration of actinomycetes can effectively reduce rat caries formation. Beneficial symbiotic bacteria of effective lactic acid bacteria and Bifidobacteria have a good effect on the treatment of porphyromonas infected gingival epithelial cells. Oral probiotics containing lactobacillus Casei and Lactobacillus rhamnosus plus multivitamin yoghurt can reduce the incidence and frequency of acute upper respiratory tract infections in women. In conclusion, the development of probiotics to regulate the pharyngeal flora of CP provides a new idea for the treatment of CP.

## 6. Conclusion

In conclusion, the abundance and community structure of pharyngeal bacteria in patients with CP changed, symbiotic beneficial bacteria tended to decrease, and the content of opportunistic pathogens increased. Therefore, to avoid overuse of antibiotics, appropriate use of probiotics will hopefully restore normal pharyngeal flora stability. At present, the 16SrDNA-based detection technology used in this study cannot determine whether the identified flora is alive at the time of sampling, which may lead to data bias. Due to the differences in the selection of sequencing fragments and bioinformatics analysis and other technical aspects, data results may eventually lead to errors. However, future metagenomic sequencing may fill in these gaps. In the future, we will further study the relationship between pharyngeal flora and CP as well as the metabolic pathways of pharyngeal flora, which will help provide new strategies for the prevention and treatment of pharyngeal diseases.

## Figures and Tables

**Figure 1:** Venn diagram of OTU analysis of pharyngeal flora of three groups (CHP, CSP, and NC).

**Figure 2:** (a) The species accumulation curve tended to be flat with the increase of sample size. (b) The dilution curve of pharyngeal flora tended to be flat with the increase of sequencing depth.

**Figure 3:** Boxplots of *α* diversity analyses.

**Figure 4:** Diagrams of principal coordinate analysis (PCoA) and *β* diversity analyses. (a) PCoA diagram of 30 samples. (b) Box plot of the species composition of three groups of bacteria. *P* < 0.05 indicates no statistical difference.

**Figure 5:** Diagrams of analysis of differences in bacterial community structure. A histogram of the composition difference of each group at phylum level (a) and at genus level (b). Bar chart of comparison of the abundance of Spirochaetes (c) and Synergistetes (d) in three groups at phylum level.

**Figure 6:** The enrichment deviation diagram of the three groups of flora distribution.

**Table 1:** OTU analysis of pharyngeal bacteria in each group.

Grouping	CHP	CSP	NC	*X*²	*P* value
Optimized sequences	55724.64 ± 1772.80	53697.73 ± 2252.19	55177.5 ± 1661.80	3.862	0.145

**Table 2:** Comparison of the relative abundance of pharyngeal flora at genus level.

	CHP	CSP	NC	*p* value
Porphyromonas	3.544 ± 2.188	1.697 ± 1.727	3.387 ± 2.002	0.042
Dialister	0.086 ± 0.085	0.016 ± 0.017	0.068 ± 0.097	0.021
*Campylobacter*	0.209 ± 0.074	0.513 ± 0.323	0.202 ± 0.204	0.006
Olsenella	0.007 ± 0.007	0.001 ± 0.002	0.003 ± 0.004	0.038
Acholeplasma	0.008 ± 0.013	0.001 ± 0.002	0	0.022
Filifactor	0.268 ± 0.21	0.033 ± 0.031	0.118 ± 0.119	0.005
TG5	0.044 ± 0.034	0.007 ± 0.012	0.017 ± 0.020	0.007
Mycoplasma	0.054 ± 0.066	0.004 ± 0.006	0.008 ± 0.006	0.001
*Escherichia*	0.003 ± 0.003	0.002 ± 0.005	0	<0.001
*Treponema*	0.443 ± 0.425	0.150 ± 0.140	0.182 ± 0.197	0.034
*Haemophilus*	5.959 ± 6.105	1.681 ± 1.740	3.560 ± 3.858	0.028
Johnsonella	0.004 ± 0.004	0.002 ± 0.001	0.002 ± 0.002	0.026
Desulfobulbus	0.003 ± 0.004	<0.001	0.001 ± 0.002	0.005
Selenomonas	0.334 ± 0.248	1.193 ± 1.124	0.448 ± 0.875	0.018
Prevotella	27.033 ± 15.260	25.064 ± 18.905	33.104 ± 13.470	0.412
Actinobacillus	0.111 ± 0.200	0.048 ± 0.086	0.448 ± 0.758	0.541

## Data Availability

The datasets used and/or analyzed during the current study are available from the corresponding author on reasonable request.
